The article "Teacher’s Emotional Intelligence and Employee Brand-Based Equity: Mediating Role of Teaching Performance and Teacher’s Self-Efficacy" was published in 2022. Journal: Front Psychol.

# Teacher’s Emotional Intelligence and Employee Brand-Based Equity: Mediating Role of Teaching Performance and Teacher’s Self-Efficacy

**DOI:** 10.3389/fpsyg.2022.901019

**Published:** 2022-05-31

**Authors:** Qiaoqiao Lu, Nor Asniza Ishak

**Affiliations:** ^1^School of Foreign Languages and Cultures, Guangdong University of Finance, Guangzhou, China; ^2^School of Educational Studies, Universiti Sains Malaysia, George Town, Malaysia

**Keywords:** teachers emotional intelligence, employee brand based equity, teaching performance, teacher’s self-efficacy, teacher – education

## Abstract

Educational institutions need to respond to global competitive problems, and branding has become a method for higher education institutions to differentiate themselves. Thus, this study attempted to investigate predictors of employee brand-based equity. A cross-sectional research design has been used to record the perception of the teachers, and data are collected using a convenience sampling technique. Before administrating the study on large scale, a pilot testing was conducted, and reliability of the scale and their items was ensured. Pilot testing results indicated a satisfactory reliability level, and constructs correlations were in the assumed directions, which allowed to conduct the study on a large scale. A sample size of 400 was set, and questionnaires were distributed among the participants, out of which, 376 were received back, while 351 were left at the end after discarding incomplete responses. The left over and completed questionnaires indicate 88% response rate. Data have been analyzed through the Smart PLS software by applying the structural equation modeling technique. After establishment of the measurement model through reliability and validity, the structural model was used to test study hypotheses. All the study hypotheses were found statistically significant on the basis of t and p statistics. Results indicate that teacher’s emotional intelligence enhances teachers’ self-efficacy, which further improves their brand-based equity. Similarly, emotional intelligence increases teacher’s performance, which also increases their brand-based equity. Limitations and future directions of the study are also reported.

## Introduction

Due to escalating competitiveness in many sectors, the themes of marketing including brand equity have gotten a lot of attention throughout the years. The actual worth of a successful brand is its capacity to capture consumer brand preference (Pinar et al., 2011) since brands reflect consumer feelings and perceptions about a brand (or service) and its performance. Furthermore, well-developed and maintained brands represent invaluable attributes and resources for businesses (Keller, 1993; Kapferer, 2004). This is due to the fact that strong brands may help businesses acquire a competitive edge (Chaharbaghi and Lynch, 1999; Kor and Mahoney, 2005) by being unique and difficult to replicate, as well as improving their financial success (Kim et al., 2003; Ponsonby-Mccabe and Boyle, 2006).

The article "Teacher’s Emotional Intelligence and Employee Brand-Based Equity: Mediating Role of Teaching Performance and Teacher’s Self-Efficacy" was published in 2022. Journal: Front Psychol.

For continuous demand and prosperity, brands should maintain their promises, generate trust, and ultimately build customer loyalty, as great brands contribute significantly to a company’s performance (Sozuer et al., 2020; Boukis et al., 2021). Among the most valuable assets for businesses is brand equity, which is a vital topic for management scholars (Christodoulides et al., 2015). “The combination of financial assets associated to a brand, company name, and logo that contribute or denounce from the value supplied by a commodity or service to a firm and/or that firm’s clients” (Kumar and Rekhi, 2018). Faced with internal and overseas competitiveness, higher education administrations have discovered that traditional or external branding initiatives are insufficient to develop strong institutional brands, as the majority of these activities appear to be centered on marketing and identification.

As a result, educational institutions began to build stronger brand strategies to respond to global competitive problems, and branding has become a method for higher education institutions to differentiate themselves (Jevons, 2006; Bunzel, 2007; Whisman, 2009). In contrast, Hemsley-Brown et al. (2016) argued that more studies are needed to gain a better knowledge of the competition and how to take advantage of the opportunities that globalization presents. Furthermore, according to Nguyen et al. (2016), a brand represents the institute’s ability to meet student demands, builds trust in its ability to supply the essential services, and aids prospective students in making the best educational and course choices. Empirical research demonstrates that, if effective, a higher education branding strategy could improve services while also attracting and retaining students (Watkins and Gonzenbach, 2013; Sultan and Wong, 2014).

Since an educational institute is a jumble of people and processes, it is difficult to discuss them apart. Current findings have deepened our awareness of the brand in the higher education context by looking into numerous challenges linked to educational institute branding (Zeithaml and Bitner, 2000; Hemsley-Brown et al., 2016). Marketing strategy has evolved into a science of branding in which both existing and future employees are targeted to achieve the corporate image promise through the promotion of a distinctive blend of direct and indirect attributes. These are work and organizational characteristics that must be unique in order for a company to obtain a competitive edge, such as employment opportunities or compensation systems (Theurer et al., 2016). All of these lead to the development of employee-based brand equity (EBBE) which is supposed to be the next new target of higher educational institutes in branding.

The article "Teacher’s Emotional Intelligence and Employee Brand-Based Equity: Mediating Role of Teaching Performance and Teacher’s Self-Efficacy" was published in 2022. Journal: Front Psychol.

According to previous studies, educating competent teaching personnel could increase educational standards. The teaching faculty at the university level is required to be dedicated to their work and take initiative. Education is widely acknowledged as the most important factor in a country’s moral, ideological, social, and economic progress. In the past two decades, countries that took big steps forward have made revolutionary achievements and performed miracles (Usarov, 2019; König et al., 2020). According to a previous study, the higher education system, particularly teachers, brings about qualitative change and enhances educational standards, guaranteeing the wellbeing, development, and growth of a country. Teachers should prepare professionally for this aim, and they must acquire capabilities at teacher training institutions (Anwer and Hussain, 2020).

For decades, organizational scientists have been trying to work out how to make a teacher successful. This intriguing subject has been studied using a variety of tactics and research methods, yet it remains unresolved. Therefore, studying teacher abilities appears to be one interesting line of inquiry that has the ability to provide answers or at the very least shed some light on the organization’s dilemma (Naderi Anari, 2012). Teacher skills are the channels through which teacher’s method, teacher’s practice, teacher’s approach, teacher’s personal qualities and teacher’s style are delivered to students to achieve effective outcomes in organizations (Gómez-Betancourt et al., 2014). All these skills are linked with emotional intelligence (EI) of the teachers, therefore, an increasing corpus of research on the role of EI for effective teachers has emerged in the past decade or two.

The belief that persons having higher levels of EI capabilities are more likely to succeed in the workplace than people who are less emotionally intelligent is at the heart of this research. Researchers have noticed that social skills are particularly important for instructors; as people move up the organizational ladder, social intelligence has become a more important factor in who will and will not succeed (Turner and Baker, 2018; Shao, 2019). Since the little investigation has been performed in an educational institutes’ context, as Kotsou et al. (2018) indicated, more solid research is needed to support the use of EI informal organizations, whether governmental or commercial, on both individual and organizational levels.

The article "Teacher’s Emotional Intelligence and Employee Brand-Based Equity: Mediating Role of Teaching Performance and Teacher’s Self-Efficacy" was published in 2022. Journal: Front Psychol.

To the best of researcher’s knowledge, no research has looked into the link between EI and EBBE in the context of educational institutions. What factors contribute to a teacher’s success in the classroom? There have been a lot of answers to this question; therefore, this question has gotten a lot of attention. Conventional indicators of competence, such as accreditation, describe less about performance, and previous attempts to enhance our understanding have generated “equivocal findings” (Rivkin et al., 2005; Klassen and Tze, 2014). Having a thorough understanding, which leads to successful teacher instruction, can influence teacher recruitment and training, as well as student performance (Corcoran, 2018). This research would keenly contribute in finding the routes for development of EBBE in educational contexts. In this way, branding strategies in higher education would also improve the level of services for students (Watkins and Gonzenbach, 2013; Sultan and Wong, 2014).

Based on the findings of Wu et al. (2018), it is assumed that teaching performance is not only an indicator of a teacher’s EI, but it could also help in developing brand equity among the teachers. Similarly, teachers’ self-efficacy could also help in developing brand equity among the teachers. To fill the gaps in previous studies, which only focused on teachers’ EI leading to their self-efficacy and performance (Wu et al., 2018), we proposed to find the role of teachers’ EI in creating employee-based brand equity in educational institutes. This research dealt with certain objectives of finding possible association between teachers’ EI and EBBE. Along with that, the author also tried to figure out the mediating roles of teaching performance and teachers’ self-efficacy toward the development of employee-based brand equity.

## Theoretical Support

Emotional intelligence has been supported by implicit theories. Individuals usually act in accordance with these theories, which act as knowledge structures by which individuals perceive themselves and others (Chiu et al., 1997; Plaks et al., 2009). As a result, implicit theories have a major impact on human behavior, and studying natural diversity within these ideas may aid in predicting how people would react to specific stimuli, therapies, or behavioral coaching. People may, for instance, hold various implicit theories about the adaptability of different cognitive, emotional, and behavioral realms of human nature (Leith et al., 2014). Intellect, emotion, interpersonal skills, relations, management skills, social judgment, and stereotyping are all examples of these realms.

The article "Teacher’s Emotional Intelligence and Employee Brand-Based Equity: Mediating Role of Teaching Performance and Teacher’s Self-Efficacy" was published in 2022. Journal: Front Psychol.

Such domains are regarded as fairly constant and complicated to change by the so-called entity sociologists. In contrast, incremental scholars see these kinds of qualities as mutable and adaptable over effort and time (Costa and Faria, 2018). Implicit intelligence theories appear to play a substantial role in behaviors and psychology of humans. People who believe in progressive theories of intelligence perceive the effort as beneficial and essential for growing ability, and they are more likely to set learning goals focused on developing their adaptable features. They are more persistent and strategic than those who believe in entity theories of intelligence, so they are more likely to create performance techniques to deal with genetic defects like puberty and the transfer from elementary to middle school (Mangels et al., 2006; Blackwell et al., 2007; Nussbaum and Dweck, 2008).

Human psychology and behavior are also heavily influenced by implicit theories of emotions. Numerous investigations with university graduates or grown-ups have found that all those who hold incremental theories about the malleability of emotions are more likely to use cognitive strategies as an emotional regulation strategy, experience more positive and fewer negative emotions, have more support networks, are more likely to use performance strategies rather than helpless strategies, and also have greater aspiration than those who hold entity theories (Burnette et al., 2012; De Castella et al., 2013). Implicit theories of emotions and intelligence are interrelated but independent; certain emotional and academic results are influenced by these, whereas others are influenced by just one.

Furthermore, numerous investigations with university graduates imply that overall emotions are more flexible than intelligence in their perspective. This is uncertain whether age and gender have an impact on implicit notions about intelligence and emotions. Several studies investigated substantial differences between women and men, while a meta-analysis produced ambiguous results (Tamir et al., 2007; Doron et al., 2009; Romero et al., 2014). This study got support from these implicit theories for evaluation of the role of EI in developing employee-based brand equity. Bandura’s (1999) interpersonal theories of self-efficacy and cognitive ability are the foundations of teachers’ self-efficacy.

Regarding social cognitive theory, self-efficacy is a critical component of human agency that “operates in harmony with other characteristics in the concept to regulate human consciousness, desire, and activity.” Both are essential for efficient operation, Bandura said that self-efficacy seems to be the essential element of human agency, the practice of self-control, and accomplishment. Believing that someone can achieve activities outside of his capability is unlikely to make it, yet, if people do not think that they own the personal potential of generating results, they will not try, regardless of if they have the potential (Bandura, 1999). So, this study also gets support from the self-efficacy theory of Bandura.

The article "Teacher’s Emotional Intelligence and Employee Brand-Based Equity: Mediating Role of Teaching Performance and Teacher’s Self-Efficacy" was published in 2022. Journal: Front Psychol.

### Teachers’ Emotional Intelligence and Employee-Based Brand Equity

People are appraised in the job based on their perceived or actual level of intelligence. In truth, a recruiter has long used intellect as a criterion when evaluating potential candidates. Although this appears to be logical, research indicates that there are additional factors to consider when recruiting great leaders and staff. Thorndike (1920) claimed that social intelligence and the capacity to get along with everyone else are extremely important for both professional and personal interactions. EI is focused on the capacity to detect one’s personal emotions, discern and classify others’ emotions, control emotions, and adapt and respond to the environment, as well as how people work together and do business tasks. Businesses have outperformed their opponents as a result of their ability to do so.

According to Goleman (1995), a top leader’s ability is to comprehend and employ EI accounts for approximately 85% of their success. If this is accurate on an interpersonal basis, organizations that nurture and use EI have a better chance of outperforming all those who do not (Goleman, 1995; Perloff, 1997). Whenever a teacher strives to control his emotions, he frequently succeeds in changing his own and others’ moods by implementing coping mechanisms that concentrate on emotion modification or resolving issues (Extremera and Fernández-Berrocal, 2008). Studies demonstrate that levels of teacher EI scores cope with unpleasant situations more constructively and are more inclined to seek positive solutions; also, teachers’ positive self-assessment in EI is linked to efficacy beliefs in reacting to students and administering the classrooms (Perry and Ball, 2007).

According to certain studies, teachers with a higher level of academic training (e.g., a doctorate) are the ones who pay the greatest attention to their students’ emotions (Soanes and Sungoh, 2019). Lee and Mamerow (2019) supported these findings, stating that individuals with greater academic qualifications also have higher values for the capacity “management of emotions in groups,” followed by those with a bachelor’s degree and then those with a master’s degree. Previously, the impact of EI of teachers has not been studied on employee-based brand equity, but it has a lot to offer as teachers are the employees of the educational institutes, and such institutes are turning into brands. It is also understood that teachers create value for their institutions (Mourad et al., 2011); therefore, we assumed that such value-creating could lead to developing brand equity in their respective institutions. We further assumed that the EI of the teachers could lead to employee-based brand equity; therefore, we suggested the following hypothesis:

***H***_1_ *: Teacher emotional intelligence is positively related to employee brand-based equity.*

The article "Teacher’s Emotional Intelligence and Employee Brand-Based Equity: Mediating Role of Teaching Performance and Teacher’s Self-Efficacy" was published in 2022. Journal: Front Psychol.

### Teachers’ Emotional Intelligence, Teachers’ Self-Efficacy, and Teachers’ Performance

One aspect that may affect teachers’ self-efficacy is EI, which measures an individual’s capacity to comprehend and regulate their emotions, as well as sympathize with and respond properly to the emotions of others (Valente et al., 2019). When assessing their level of self-efficacy, teachers look at their own teaching abilities (Tschannen-Moran et al., 1998; Sutton and Wheatley, 2003). Teaching competency varies depending on the teaching activity; however, all teaching tasks require the ability to work with emotion. Teachers must regulate, evaluate, and manage their emotions in order to achieve pedagogical efficacy and create a happy learning environment (Gates, 2000). Therefore, regardless of the teaching task, teachers are likely to include their EI when assessing their level of self-efficacy (Wu et al., 2018).

Emotional intelligence is strongly connected with instructors’ sense of self-efficacy, according to empirical findings. EI components may also influence teachers’ self-efficacy (Sarkhosh and Rezaee, 2014). Chan (2004) discovered that secondary school teachers in Hong Kong’s empathic sensitivity predicted self-efficacy toward assisting others, and also that positive emotion control impacted overall self-efficacy. Social and emotional competence, as per the prosocial classroom approach, can assist instructors in achieving good performance. Teachers with a high level of social and emotional competence, in particular, are better at using emotions and verbal assistance to encourage students’ passion for learning and to lead and manage student behavior (Chan, 2004).

Furthermore, these teachers have a better awareness of the mechanisms of instructional situations of conflict, resulting in a significant reduction in disruptive behavior. Teachers having greater EI seem to have superior teaching performance, according to the empirical data (Yoke and Panatik, 2015). In conclusion, past research has shown that EI has an impact on teaching performance and is linked to teachers’ self-efficacy perceptions. EI, according to Sarkhosh and Rezaee (2014), improves teachers’ performance accomplishment, which in turn contributes to better self-efficacy (Wu et al., 2018). As a result, we looked into the relationships between EI, instructional effectiveness, and instructors’ self-efficacy. We hypothesized that because instructors with higher EI have better teachers’ performance, their confidence and self-efficacy will be shaped by this:

***H***_2_ *: Teacher emotional intelligence is positively related to employee teacher’s self-efficacy.*

The article "Teacher’s Emotional Intelligence and Employee Brand-Based Equity: Mediating Role of Teaching Performance and Teacher’s Self-Efficacy" was published in 2022. Journal: Front Psychol.

***H***_3_ *: Teacher emotional intelligence is positively related to teaching performance.*

### Mediating Role of Teachers’ Self-Efficacy and Teaching Performance

The essential characteristics of human freedom expressed as effort and perseverance devoted to the achievement of the goals are captured by a people’s self-efficacy, which functions as an intrapersonal incentive factor. Teachers’ self-efficacy was being demonstrated to affect their teaching techniques, passion, dedication, and teaching behaviors, as well as their tenacity in dealing with problematic learners (Skaalvik and Skaalvik, 2007). However, no motivating component has unchanging impacts, including situational circumstances, tools to generate validity, and self-appraisal precision all influence self-efficacy (Bandura, 2011).

Emotional intelligence is positively correlated with or anticipates teachers’ self-efficacy. Fabio and Palazzeschi (2008) employed a multiple regression model to investigate the relationship between self-efficacy and EI in an Italian teacher’s research. Increased EI was found to be linked to higher self-efficacy in three different categories (i.e., educational approaches, student participation, and classroom organization). Furthermore, the intrapersonal dimension of EI was found to be a superior predictor of all three dimensions of instructors’ self-efficacy (Alrajhi et al., 2017). A lot of investigations indicated that EI proved to be the predictor of teachers’ self-efficacy (Yazici et al., 2011; Gharetepeh et al., 2015; Black et al., 2019; Pérez-Fuentes et al., 2019; Valente et al., 2020).

A few researchers also evaluated the mediating role of teachers’ self-efficacy in various contexts (Shaterian Mohamadi and Asadzadeh, 2011; Kunemund et al., 2020). These findings suggested that teachers’ self-efficacy could be utilized as a mediator between teachers’ EI and EBBE in this research. Inputs, procedures, and outputs can be used to evaluate a teacher’s performance. Most of the studies on “teacher performance” provide a sense of direction or the instructor’s impact on student accomplishment. Although it is possible that the best way to assess teacher performance is to look at increases in a diverse selection of student learning, such as academic and social outcomes, it is also possible that the best way to assess teacher performance is to look at increases in a variety of different types of student learning (Corcoran and Tormey, 2013).

The article "Teacher’s Emotional Intelligence and Employee Brand-Based Equity: Mediating Role of Teaching Performance and Teacher’s Self-Efficacy" was published in 2022. Journal: Front Psychol.

Emotional intelligence is thought to be the foundation for emotionally smart and interpersonally suitable teaching approaches (Corcoran and Tormey, 2013). Furthermore, we are currently unaware of any scientific findings that would allow us to determine if greater amounts of assessed EI are linked to more successful teacher performance in establishing the EBBE. In reality, among working teachers, there is very less data on EI (Corcoran and Tormey, 2013). A few researchers recently evaluated the impact of EI on teaching performance (Wahyudi, 2018; Kaur et al., 2019; Akhtar et al., 2020), but they did not check their impacts on EBBE. A few also evaluated the mediating role of teaching performance between EI and teachers’ self-efficacy (Wu et al., 2018). This literature about the interconnectedness of EI with teachers’ self-efficacy and teaching performance allowed us to suggest the following hypotheses:

***H***_4_ *: Teacher’s self-efficacy mediates the relationship of teacher emotional intelligence and employee brand-based equity.*

***H***_5_ *: Teaching performance mediates the relationship of teacher emotional intelligence and employee brand-based equity.*

The conceptual model (Figure 1) has been formed based on the above literature and hypotheses.

**FIGURE 1:** Conceptual framework.

## Participants and Procedure

This study used a cross-sectional research design to record the perception of the teachers. In the past studies, the usage of cross-sectional research design is common and prevalent (Wu et al., 2018); thus, this study has utilized this research design. We have used the survey research method, and data are collected using a convenience sampling technique. A convenience sampling technique comes under the domain of non-probability sampling technique, and its application in survey-based research is common, and previous researchers have used it frequently (Ali et al., 2015; Saqib et al., 2017). A convenience sampling technique provides an ease and access in terms of cost and time in data collection. Hence, perception of teachers was obtained in this study through this sampling technique. In the past, other studies have also used teachers as target population in previous studies (e.g., Abun, 2021).

The article "Teacher’s Emotional Intelligence and Employee Brand-Based Equity: Mediating Role of Teaching Performance and Teacher’s Self-Efficacy" was published in 2022. Journal: Front Psychol.

In this regard, administration of the academic institutes was requested to accord formal approval to collect data from the teaching staff. After getting prior approval from the administration, a list of faculty members along with their contact details was obtained, and later, teaching staff was approached for data collection on the basis of available contact lists. They were briefed about the study and its intended outcomes. Moreover, written informed consent was obtained from the participants. Before administrating study on a large scale, a pilot testing was conducted, and reliability of the scales and their items was ensured. Pilot testing results indicated a satisfactory reliability level, and constructs correlations were in the assumed directions, which allowed us to move forward for large-scale data collection.

A reasonable and suitable sample size was devised based on the recommendations of available literature (Krejcie and Morgan, 1970) and previously used by Bashir et al. (2019, 2020) and Wu et al. (2022). Keeping in view the recommendations, a sample size of 384 was sufficient; hence, we set a benchmark of 400 as sample size and floated questionnaire among the teaching staff of academic institutes. Out of these 400 distributed questionnaires, 376 were received back. After discarding the incomplete responses, the useable questionnaires were left as 351, which have been used for the data analysis purpose. Thus, the response rate remained at 88%, which is sufficient in cross-sectional survey-based research.

Issues of common method bias can shatter the results in cross-sectional research; thus, we employed various techniques to address this issue; first, we used reverse-coded questions/scale items to restrict respondents from providing monotonic responses. Second, we have interchanged the position of variables in the questionnaires, so that respondents could not develop a correlation. Finally, we ensured respondents that collected data will be used only for academic purpose, and their feedback will be strictly kept under confidentiality (Bashir et al., 2019, 2020).

First part of the questionnaire was related to the demographic features of the teaching staff related to their age, gender, and teaching experience along with their academic qualification. Demographic statistics indicate that majority of the respondents have 18 years of education, while respondents having age above 25 years occupy major composition in the participants. Similarly, almost equal number of respondents were single (48%) and married (52%) with minor differences in proportion. Similar patterns were observed in case of gender, and male and female teaching staff was almost equally distributed in sample respondents.

The article "Teacher’s Emotional Intelligence and Employee Brand-Based Equity: Mediating Role of Teaching Performance and Teacher’s Self-Efficacy" was published in 2022. Journal: Front Psychol.

### Scales/Measurement

We have used a 5-point Likert scale (i.e., 5–1), where 5 indicates a situation of strongly agree and 1 indicates a situation of strongly disagree. The independent variable (teachers’ EI) of this study is operationalized on the basis of 15-item Teachers’ Emotional Competence Scale (Wu et al., 2018). The original version of this scale consists of six dimensions and total of twenty four items. However, we have conceptualized most relevant dimensions of this scale and adapted fifteen items from this scale, covering the dimensions of self-emotion awareness (SEA) with four items, self-emotion regulation (SER) with four items, students’ emotion identification (SEI) with four items, and students’ emotion management (STEM) with three items. Sample items for this scale includes, “I do not pay much attention to students emotions in class” (reverse coded) and “I have the ability to influence students’ emotions.”

Similarly, a mediating variable, teaching performance was measured on the basis of four items previously used by Corcoran and Tormey (2013) and Wu et al. (2018). Sample items include, “I seriously monitor students in class to prevent disruptive behavior,” and we have used one dimension of this scale relevant to our conceptualization. The other mediating variable of this study, i.e., teacher’s self-efficacy is the measure on the basis of scale developed by Yu et al. (1995) through the Teachers’ Sense of Teaching Efficacy Scale (TSTES). The sample item for this scale includes, “I can change students with learning disabilities if I work hard.” We have conceptualized the personal teaching efficacy (PTE) dimension of this scale. Finally, EBBE is measured on the basis of five items of Baumgarth and Schmidt (2010). Sample statement of this scale includes, “I am aware that everything I say or do can affect the brand image.” We have used reverse-coded items in the scale to restrict the respondents from providing monotonic responses.

## Results

### Assessment of Measurement and Structural Model

We have opted a multivariate data analysis tool to test the hypothesized relationships of this study. For this purpose, structural equation modeling (SEM) is performed using Smart PLS 3.9 (Ali et al., 2018; Bashir et al., 2020). Owing to several reasons, we have used Smart PLS; it is highly comfortable with complicated models and can handle tiny samples quickly (Hair et al., 2016). Furthermore, it has the capacity to handle non-normal data with ease, and non-parametric data are simply handled, and finally, it can be used where theory is less developed. The conceptualized model of this study is termed as where theory pertaining to EBBE is less developed. So, based on these issues, the usage of Smart PLS was a good available option. SEM is evaluated in two ways, i.e., one for measurement model evaluation and the other for structural model evaluation (Hair et al., 2019).

The article "Teacher’s Emotional Intelligence and Employee Brand-Based Equity: Mediating Role of Teaching Performance and Teacher’s Self-Efficacy" was published in 2022. Journal: Front Psychol.

The measuring model was evaluated for its reliability and validity. For this purpose, alpha, rho-a, and composite reliability (CR) were assessed, and it was observed that all the indicators of reliability are above the threshold value, i.e., >0.60. These indicators are indicating a good level of reliability. In this regard, the value of alpha for EBBE was 0.744, and the highest value of alpha was observed for the construct teachers’ EI, i.e., 0.931 (Hair et al., 2011; Bashir et al., 2020). Other parameters of reliability, i.e., rho-A and composite reliability were also within the acceptable limit.

To test the convergent validity, we have used two measures, namely, one is average variance extracted (AVE) and second is outer loadings. Results indicate that AVE of the respective constructs was above the requited limit of 0.50, which indicates that convergent validity has been established (Mela and Kopalle, 2002).

In case of outer loadings (Figures 2, 3, and Table 1), the values of the outer loadings were within the acceptable limits, i.e., >0.708; however, some values were observed low as compared with the benchmark. Values less than 0.40 were dropped from further analysis; however, some values with lower outer loadings have been retained in this study because AVE of the respective construct was within the acceptable range (>0.50). In this regard, one item in EBBE has lower overloading, while two items from teacher’s EI and one item from teacher performance have lower outer loadings. However, the AVE of the respective construct was higher than the limit. While talking about the droppage of items from construct, one item has been dropped from EBBE (EBBE-3) and one item from teachers’ self-efficacy (TSE-2) has also been dropped. No item has been dropped from teacher’s performance, while four items have been dropped from teacher’s EI scale (i.e., TEI-3, TEI-10, TEI-11, and TEI-15) due to very low outer loadings.

**FIGURE 2:** Path estimates.

**FIGURE 3:** Path significance.

**TABLE 1:** Reliability and convergent validity of the study constructs.

Construct	Indicator	FL	VIF	Cronbach’s Alpha	rho_A	Composite reliability	AVE
EBBE	BE1	0.761	1.215	0.744	0.767	0.830	0.550
	BE2	0.687	2.070				
	BE4	0.761	1.419				
	BE5	0.755	2.327				
TEI	TEI1	0.771	2.118	0.931	0.940	0.942	0.596
	TEI12	0.777	3.580				
	TEI13	0.763	3.792				
	TEI14	0.735	3.203				
	TEI2	0.877	4.673				
	TEI4	0.796	3.636				
	TEI5	0.630	1.545				
	TEI6	0.861	3.567				
	TEI7	0.676	1.809				
	TEI8	0.816	4.869				
	TEI9	0.757	3.424				
TP	TP1	0.654	1.381	0.835	0.869	0.891	0.675
	TP2	0.790	1.774				
	TP3	0.927	5.525				
	TP4	0.889	4.756				
TSE	TSE1	0.914	2.856	0.884	0.975	0.918	0.738
	TSE3	0.945	4.534				
	TSE4	0.787	2.071				
	TSE5	0.779	1.990				

*TEI, teacher’s emotional intelligence; EBBE, employee brand-based equity; TSE, teacher’s self-efficacy; TP, teacher’s performance.*

The article "Teacher’s Emotional Intelligence and Employee Brand-Based Equity: Mediating Role of Teaching Performance and Teacher’s Self-Efficacy" was published in 2022. Journal: Front Psychol.

We have used very well-established criteria to assess discriminant validity (Table 2), i.e., HTMT ratios (Hair et al., 2016). Two tables, Table 3 (Fornell and Larcker criteria) and Table 4 (HTMT ratios), in this regard indicate establishment of discriminant validity. The square root of the AVE of variables is larger than the correlations among them, according to the first condition (Hair et al., 2011), which offsets the first criteria and establishes discriminant validity.

**TABLE 2:** Discriminant validity (Fornell-Larcker-1981 Criteria).

Construct	EBBE	TEI	TP	TSE
EBBE	***0.742***			
TEI	0.676	***0.772***		
TP	0.485	0.318	***0.822***	
TSE	0.478	0.294	0.351	***0.859***

*TEI, teacher’s emotional intelligence; EBBE, employee brand-based equity; TSE, teacher’s self-efficacy; TP, teacher’s performance. The bold values are indicate the results for corresponding statistics for whole variable not the items.*

**TABLE 3:** Discriminant validity (HTMT).

Construct	BE	TEI	TP	TSE
BE	–	–	–	–
TEI	0.691	–	–	–
TP	0.606	0.359	–	–
TSE	0.564	0.300	0.392	–

*TEI, teacher’s emotional intelligence; EBBE, employee brand-based equity; TSE, teacher’s self-efficacy; TP, teacher’s performance.*

**TABLE 4:** Direct, indirect, and total path estimates.

Direct path	Beta	SD	*t*	*p*
TEI - > EBBE	0.532	0.040	13.336	**0.000**
TEI - > TP	0.318	0.056	5.679	**0.000**
TEI - > TSE	0.294	0.055	5.302	**0.000**
TP - > EBBE	0.231	0.049	4.730	**0.000**
TSE - > EBBE	0.240	0.038	6.356	**0.000**
**Specified indirect path**				
TEI - > TSE - > EBBE	0.071	0.017	4.147	**0.000**
TEI - > TP - > EBBE	0.073	0.020	3.674	**0.000**
**Total indirect path**				
TEI - > BE	0.144	0.027	5.272	**0.000**
**Total path**				
TEI - > EBBE	0.676	0.029	23.392	**0.000**

*TEI, teacher’s emotional intelligence; EBBE, employee brand-based equity; TSE, teacher’s self-efficacy; TP, teacher’s performance. The bold values are indicate the results for corresponding statistics for whole variable not the items.*

Similarly, another way for evaluating discriminant validity has been used as assessment of HTMT. As long as the HTMT ratios in all columns are less than 0.90 and 0.85, both liberal and conservative HTMT benchmarks have been met (Table 4).

The article "Teacher’s Emotional Intelligence and Employee Brand-Based Equity: Mediating Role of Teaching Performance and Teacher’s Self-Efficacy" was published in 2022. Journal: Front Psychol.

In addition to these measures, we have used other established criteria to test the model fitness, i.e., coefficient of determination (R^2^) and effect size (f^2^). The effect size was found to be good and acceptable, i.e., larger than 0.01 (Hair et al., 2006; Bashir et al., 2020). While in case of coefficient of determination, it can be said that good effect size has been observed; first, Figure 2 illustrates that 8% change in teacher’s self-efficacy is being observed through teachers’ EI, while 11% change is being observed in teaching performance through teacher’s EI (Figure 2). Predictor and mediating variables (both) collectively explain 56% change in EBBE (Hair et al., 2016). Predictive relevance (Q^2^) of the model is observed satisfactory as value of Q^2^ has been observed larger than zero (Geisser, 1975).

### Hypotheses Testing

Hypotheses testing in this study is carried out on the basis of path estimates; in this regard, p and t statistics have been inspected. Table 4 depicts/illustrates path estimation, while Table 5 illustrates hypotheses testing. H1, i.e., teachers’ EI is positively related to EBBE, has been proved statistically significant (*t* > 1.96 and *p* < 0.05). The value of coefficient in this regard is 0.532, which indicates that one unit change in teacher’s EI will bring 0.532 unit change in EBBE. Thus, H1 is supported. Similarly, second hypothesis (H2) of this study, i.e., teacher’s EI is positively related to teacher’s self-efficacy, and it has also been statistically proved, which indicates that teacher’s EI promotes teacher’s self-efficacy. This argument is supported through *p* and *t* statistics (*t* > 1.96 and *p* < 0.05), and the value of beta in this regard indicates that one unit change in teachers’ EI will bring 0.294 units change in teachers’ self-efficacy, providing an evidence that H2 is supported. Similarly, H3 of this study, which is related to teachers’ EI, is positively related to teaching performance and is also statistically proved on the basis of *t* and *p* statistics. Both the parameters of hypothesis testing are met. Thus, H3 is supported. The last two hypotheses are related to the mediation effect, and these two are also supported through the statistical evidence as indirect effect in both cases is found statistically significant (*t* > 1.96 and *p* < 0.05). Specified indirect effect in both cases is almost equal and statistically significant. Hence, both H4 and H5 are supported. Thus, it can be argued that teachers’ EI promotes teachers’ self-efficacy, which further improves the EBBE. Similarly, teacher’s EI increases teacher’s performance, which further increases EBBE.

The article "Teacher’s Emotional Intelligence and Employee Brand-Based Equity: Mediating Role of Teaching Performance and Teacher’s Self-Efficacy" was published in 2022. Journal: Front Psychol.

**TABLE 5:** Hypotheses testing.

Hypotheses		Coefficient (Beta)	S.D.	*t*	*p*	Status
H1	TEI - > EBBE	0.532	0.040	13.336	0.000	Supported
H2	TEI - > TSE	0.294	0.055	5.302	0.000	Supported
H3	TEI - > TP	0.318	0.056	5.679	0.000	Supported

**Mediation hypotheses**											

H4	TEI - > TSE - > EBBE	0.071	0.017	4.147	0.000	Supported
H5	TEI - > TP - > EBBE	0.073	0.020	3.674	0.000	Supported

*TEI, teacher’s emotional intelligence; EBBE, employee brand-based equity; TSE, teacher’s self-efficacy; TP, teacher’s performance.*

## Discussion

This research focused on developing a sense of branding in educational institutions. As suggested by Mourad et al. (2011), it is possible to develop brand equity in higher education, and to our understanding, teachers are the employees of educational institutes, which could be a part of EBBE. Therefore, this study was designed and conducted. The aspects, associated with teachers such as their EI, self-efficacy, and performance, were assessed based on the suggestions of previous investigations such as Wu et al. (2018). The research provided notable insights into the previously unexplored dimension of EBBE development in educational institutes. Some direct, as well as indirect, relationships between these factors were studied in the research.

The major direct relationship between teachers’ EI and EBBE proved that intelligence associated with the emotions of the teachers is a strong predictor of EBBE in educational institutes. This is supported by the fact that EI provides the support to individuals to cope with any kind of circumstances (Naderi Anari, 2012; Wu et al., 2018). While teachers are the employees of educational institutions, they are more concerned with the results of their students. Once their students get good grades, they are automatically charged up for doing more dedicated efforts in future. All this comes through their EI. This helps in developing brand equity for the respective organization as well. Previously, no research has been conducted in this regard.

The other direct relationships of EI with teachers’ self-efficacy and teaching performance have also been studied in this research. The results indicated that teachers’ EI was strongly associated with their self-efficacy and performance. This happens because EI bridges the association of lacking motivation in teachers for doing their best. Previously, some researchers found that EI of teachers was significantly affecting their self-efficacy (Yazici et al., 2011; Gharetepeh et al., 2015; Black et al., 2019; Pérez-Fuentes et al., 2019; Valente et al., 2020). This suggests that educators with higher levels of EI are more efficacious in their job. The obtained result was consistent with the conclusions of Sarkhosh’s investigations (Sarkhosh and Rezaee, 2014). At higher educational institutions and language institutes, these studies found a favorable relationship between teachers’ EI and self-efficacy.

The article "Teacher’s Emotional Intelligence and Employee Brand-Based Equity: Mediating Role of Teaching Performance and Teacher’s Self-Efficacy" was published in 2022. Journal: Front Psychol.

Furthermore, the outcome backs up Chan’s findings (Chan, 2004). Teachers in primary and secondary schools showed a strong relationship between EI and self-efficacy, according to these studies. Considering the findings of several studies on EI and teacher efficacy, as well as the conclusions of this study, it can be concluded that the aspect of teachers’ self-efficacy is crucial and significant, irrespective of the academic settings in which they teach. Keeping it precise, it is understood that no matter where the teacher is teaching, their EI leads to self-efficacy. The results of this study are also in agreement with some of the scholars who found strong association between EI and teaching performance (Wahyudi, 2018; Kaur et al., 2019; Akhtar et al., 2020). These results are clearly indicating that if EI of teachers is considered efficiently then their performance improves.

The indirect effects of teachers’ self-efficacy were also tested in this study between teachers’ EI and EBBE. The results provided support for mediating the role of teachers’ self-efficacy in this relationship. Although the direct effects were also significant, it proved that if teachers were more self-efficacious in their teaching, then it could enhance the association of EI with EBBE. Hence, it strengthened our notion that the EI of teachers could predict EBBE in their institutions. Previously, teachers’ self-efficacy was considered to affect the techniques of teachers, their passion, dedication to instruct, and behaviors, as well as their ability in dealing with challenging students (Skaalvik and Skaalvik, 2007). Some of the past researchers also found significant mediation of teachers’ self-efficacy in different perspectives (Shaterian Mohamadi and Asadzadeh, 2011; Kunemund et al., 2020).

The last hypothesis was about mediating role of teaching performance of the teachers between teachers’ EI and EBBE. The results proved that if teaching performance becomes the target of teachers in the sense of competing with other teachers at their workplace, then it could lead to the sense of competition. Due to this kind of competition, teachers are more motivated to prove their worth. The EI of such teachers helps them in doing their best among others. Although the role of EI in having a positive impact on EBBE development is also significant in this research, teaching performance proved that such a task-oriented dimension of teaching could enhance the relationship of EI with EBBE. Previously, few researchers indicated that EI leads to improved teaching performance (Wahyudi, 2018). Some of the scholars indicated that EI, teachers’ self-efficacy, and teaching performance are interconnected factors (Wu et al., 2018), and teaching performance was used as a mediator in their studies.

The article "Teacher’s Emotional Intelligence and Employee Brand-Based Equity: Mediating Role of Teaching Performance and Teacher’s Self-Efficacy" was published in 2022. Journal: Front Psychol.

## Conclusion

On the basis of available empirical evidence of this study, it can be concluded that teacher’s EI has the potency to improve the teacher’s teaching performance. Similarly, emotionally intelligent teachers improve their self-efficacy, which becomes a source to enhance their teaching performance. Moreover, teachers with high EI improve their commitment level, and they become more loyal and ambassadors of their organizations when their brand-based equity is established. Thus, organizations should focus on improving the EI of their teaching staff so that their teaching performance and self-efficacy could be improved. Teachers with high emotional intelligent can promote a constructive competition at workplace, which can be helpful for other teachers to increase their performance to compete others. This can trigger teachers to get more motivated to prove their worth. Empirical evidence of this study indicates that teachers’ EI promotes teachers’ self-efficacy, which develops EBBE. Similarly, teacher’s EI increases teacher’s performance, which further increases EBBE, and employees perceive a sense of pride to be a part of the organization.

## Theoretical and Practical Implications

From the theoretical perspective, this study has touched the boundaries of EBBE and made an attempt to extend the body of knowledge related to EBBE. Thus, this study contends to add into the knowledge stream of EBBE, teacher’s performance, and teacher’s EI. This study established that EI has the tendency to develop EBBE, which is a unique contribution into the existing body of knowledge. Second, this study tests mediating role of teachers’ self-efficacy between the relationship of teachers’ EI and EBBE; third, this study also established a mediating role between the relationship of teachers’ EI and EBBE, which is also a contribution of this study. From the practical point of view, this study contends that practitioners should focus on developing EI of the teaching staff and should provide them trainings to enhance their EI. It will promote their self-efficacy, and higher self-efficacy is attached with positive outcomes, so teachers with higher self-efficacy will show positive behaviors at workplace, which will be beneficial for the academic institutes. Additionally, it will promote teachers’ performance too.

## Limitations of the Study

Just like other studies, this study has also some limitations. First, this study used a cross-sectional research design, which does not allow drawing a cause and effect relationship. So, in future studies, researchers should focus on the longitudinal research design. Second, we have collected data using the convenience sampling technique, so in future, other probability sampling techniques should be used to collect data for improved and deeper insights. We have used the non-parametric data analysis tool, thus using the parametric data analysis tool in future can provide interesting outcomes. Additionally, we have used a mediating phenomenon through teacher’s self-efficacy and teaching performance, so in future, other possible mediators can also be used. In this regard, job satisfaction can be a potential mediator. Similarly, the moderating phenomenon such as supervisor’s support, organizational support, and prevalence of ethical climate can also be used as potential moderators of the study. Similarly, it would be interesting to split EBBE and brand allegiance, brand endorsement, and brand consistent behavior should be checked in future studies. Moreover, in future studies, comparison of perception of college and university teachers could provide deeper insights.

The article "Teacher’s Emotional Intelligence and Employee Brand-Based Equity: Mediating Role of Teaching Performance and Teacher’s Self-Efficacy" was published in 2022. Journal: Front Psychol.

## Data Availability Statement

The original contributions presented in the study are included in the article/supplementary material, further inquiries can be directed to the corresponding author.

## Ethics Statement

This study was reviewed and approved by Shanghai University of Finance and Economics (SUFE), Shanghai, China. Written informed consent was obtained from all participants for their participation in this study. The study was conducted in accordance with the Declaration of Helsinki.

## Author Contributions

QL drafted the final manuscript. NI did analysis and proofread. Both authors contributed to the article and approved the submitted version.

## Conflict of Interest

The authors declare that the research was conducted in the absence of any commercial or financial relationships that could be construed as a potential conflict of interest.

## Publisher’s Note

All claims expressed in this article are solely those of the authors and do not necessarily represent those of their affiliated organizations, or those of the publisher, the editors and the reviewers. Any product that may be evaluated in this article, or claim that may be made by its manufacturer, is not guaranteed or endorsed by the publisher.
